The article "Integrated Analysis of Circular RNA-Associated ceRNA Network Reveals Potential circRNA Biomarkers in Human Breast Cancer" was retracted in 2023. Reasons: signs of a paper mill; suspected computer-generated content; unreliable results or conclusions; concerns about the data.

# Integrated Analysis of Circular RNA-Associated ceRNA Network Reveals Potential circRNA Biomarkers in Human Breast Cancer

**DOI:** 10.1155/2021/1732176

**Published:** 2021-12-20

**Authors:** Han Sheng, Huan Pan, Ming Yao, Longsheng Xu, Jianju Lu, Beibei Liu, Jianfen Shen, Hui Shen

**Affiliations:** ^1^Department of Nursing, The First Affiliated Hospital of Jiaxing University, Jiaxing 314000, China; ^2^Department of Central Laboratory, The First Affiliated Hospital of Jiaxing University, Jiaxing 314000, China; ^3^Department of Anesthesiology and Pain Medicine, The First Affiliated Hospital of Jiaxing University, Jiaxing 314000, China; ^4^Department of Breast Disease, The First Affiliated Hospital of Jiaxing University, Jiaxing 314000, China

## Abstract

Circular RNA (circRNA) is closely related to tumorigenesis and cancer progression. Yet, the roles of cancer-specific circRNAs in the circRNA-related ceRNA network of breast cancer (BRCA) remain unclear. The aim of this study was to construct a ceRNA network associated with circRNA and to explore new therapeutic and prognostic targets and biomarkers for breast cancer. We downloaded the circRNA expression profile of BRCA from Gene Expression Omnibus (GEO) microarray datasets and downloaded the miRNA and mRNA expression profiles of BRCA from The Cancer Genome Atlas (TCGA) database. Differentially expressed mRNAs (DEmRNAs), differentially expressed miRNAs (DEmiRNAs), and differentially expressed circRNAs (DEcircRNAs) were identified, and a competitive endogenous RNA (ceRNA) regulatory network was constructed based on circRNA–miRNA pairs and miRNA–mRNA pairs. Gene ontology and pathway enrichment analyses were performed on mRNAs regulated by circRNAs in ceRNA networks. Survival analysis and correlation analysis of all mRNAs and miRNAs in the ceRNA network were performed. A total of 72 DEcircRNAs, 158 DEmiRNAs, and 2762 DE mRNAs were identified. The constructed ceRNA network contains 60 circRNA–miRNA pairs and 140 miRNA–mRNA pairs, including 40 circRNAs, 30 miRNAs, and 100 mRNAs. Functional enrichment indicated that DEmRNAs regulated by DEcircRNAs in ceRNA networks were significantly enriched in the PI3K-Akt signaling pathway, microRNAs in cancer, and proteoglycans in cancer. Survival analysis and correlation analysis of all mRNAs and miRNAs in the ceRNA network showed that 13 mRNAs and 6 miRNAs were significantly associated with overall survival, and 48 miRNA–mRNA interaction pairs had a significant negative correlation. A PPI network was established, and 21 hub genes were determined from the network. This study provides an effective bioinformatics basis for further understanding of the molecular mechanisms and predictions of breast cancer. A better understanding of the circRNA-related ceRNA network in BRCA will help identify potential biomarkers for diagnosis and prognosis.

## 1. Introduction

Breast cancer is one of the most common cancers among women worldwide [1], with strong invasiveness and a high incidence of metastasis [2]. Currently, breast cancer treatments include surgery, radiation therapy, endocrine therapy, chemotherapy, and biotargeted therapy. However, the recurrence rate and drug resistance in some patients are still high, and the therapeutic effect and prognosis of breast cancer are not satisfactory. Therefore, breast cancer's molecular pathogenesis needs to be further explored, and the identification of new candidate therapeutic targets and biomarkers is urgently needed.

Bioinformatics analysis has been widely applied in oncology to identify genetic changes and new potential biomarkers associated with cancer [3]. In the past few decades, 70%-90% of the transcribed human genome has been searched. Related data indicate that protein-coding genes account for only about 2% of the human genome, and noncoding RNAs make up the majority of the human transcriptome [4]. Noncoding RNAs, including circular RNAs (circRNAs), microRNAs (miRNAs), long nocoding RNAs (lncRNAs), and small nuclear RNAs, are a large class of RNA molecules that do not encode proteins but may regulate specific functions in the cells. The competitive endogenous RNA (ceRNA) hypothesis reveals a new mechanism for interaction between RNAs. The main idea of the ceRNA hypothesis is that multiple types of RNA transcripts communicate with each other by competing for binding to shared miRNA-binding sites (miRNA response elements or MREs) [5].

circRNA is a class of covalently closed single-stranded circular RNA molecules without free 5 or 3 end, which makes them well expressed and more stable than their linear counterparts. circRNAs contain multiple miRNA-binding sites that bind to miRNAs, which are seen as miRNA sponges that inhibit miRNA activity and regulation of expression of their downstream target genes [6, 7]. circRNA, which is abundant in eukaryotic cells, highly conserved, and structurally stable, has certain tissue, time, and disease specificity. Due to these characteristics, circRNA has become a new focus of research [8].

A number of circRNAs have been discovered in various cancers where they can be activated, inhibiting tumor progression or promoting tumorigenesis. For example, circ-MTO1 can inhibit the progression of liver cancer cells [9]. circ-LARP4 can inhibit cell proliferation and invasion of gastric cancer cells by sponging miR-424-5p and regulating the expression of LATS1 [10]. circ-FBXW7 suppresses glioma development, while its expression is positively correlated with the overall survival of patients with glioblastoma [11]. The hsa_circ_001783 regulates breast cancer (in vitro) by sponging miR-200c-3p to regulate ZEB1/2 and ETS1 and is associated with poor clinical outcomes in breast cancer patients [12].

In the current study, we collected the expression profiles of circRNA, miRNA, and mRNA from BRCA tissues and adjacent normal mammary gland tissues from the Gene Expression Omnibus (GEO) database and The Cancer Genome Atlas (TCGA) database. We performed a comprehensive analysis of these expression profiles to identify differentially expressed mRNAs (DEmRNAs), differentially expressed miRNAs (DEmiRNAs), and differentially expressed circRNAs (DEcircRNAs). After predicting the sponging of miRNAs by circRNA and miRNA target genes, we constructed a circRNA-miRNA-mRNA network. To investigate the main functional pathways involved in the development of breast cancer in this ceRNA network, DEmRNAs of the ceRNA network were assessed by gene ontology (GO) annotation and Kyoto Encyclopedia of Genes and Genomes (KEGG) pathway analyses. A protein-protein interaction network was also established. Finally, we performed an overall survival analysis of miRNAs and mRNAs in ceRNA networks to identify prognostic biomarkers associated with breast cancer. This study furthers the understanding of molecular mechanisms underlying breast cancer development and provides potential circRNA, miRNA, and mRNA biomarkers for the early diagnosis, treatment, and prognosis of breast cancer.

## 2. Materials and Methods

### 2.1. Expression Profiling in the Cancer Genome Atlas and Gene Expression Omnibus

The mRNA and miRNA sequence data of breast cancer were extracted from the TCGA database (https://portal.gdc.cancer.gov/). All file data were downloaded using the GDC Data Transfer Tool (Provided by GDC Apps) (https://tcga-data.nci.nih.gov/). The mRNA profiles contained 1097 BRCA tissues and 114 adjacent normal tissues, and the miRNA profiles contained 1092 BRCA tissues and 105 adjacent normal tissues. The exclusion criteria were samples without clinical data and samples without complete information of stage and overall survival period.

The circRNA expression profiles of BRCA were downloaded from GEO database (http://www.ncbi.nlm.nih.gov/geo) by searching keywords ((“breast neoplasms” (MeSH Terms) OR breast cancer (All Fields)) AND circRNA (All Fields)) AND (“Homo sapiens” (Organism) AND (“Non-coding RNA profiling by array” (Filter) OR “Non-coding RNA profiling by high throughput sequencing” (Filter))). We selected data according to the following criteria: selected datasets should be circRNA transcriptome data of the whole genome. These data were derived from tumor tissues and adjacent normal tissues of patients with BRCA, and datasets were standardized or raw datasets. The GSE101123 dataset met the screening requirements and was used in this study. The dataset included 3 normal mammary gland tissues and 8 BRCA tissues. These expression profiles did not require ethical approval or informed consent as they were publicly available data from TCGA and GEO.

### 2.2. Identification of Differentially Expressed mRNAs, miRNA, and circRNA in Breast Cancer Compared to Adjacent Tissues

Firstly, mRNAs/miRNAs detected with difficulty, which showed read count value = 0 in more than 50% samples, were filtered and deleted. To obtain the differentially expressed mRNAs (DEmRNAs) and miRNAs (DEmiRNAs) between normal tissues and BRCA, the count data were processed with the Bioconductor package edge R software [13]. All RNA expression levels were standardized to the sample mean. The *P* value was corrected with a false discovery rate (FDR). The threshold for the expression of DEmRNAs and DEmiRNAs was FDR < 0.01 and ∣log_2_fold change | >1. Additionally, the differently expressed circRNAs (DEcircRNAs) were screened using the limma package. The threshold for the expression of DEcircRNAs was *P* value < 0.01 and ∣log_2_fold change | >1.

### 2.3. Construction of the ceRNA Regulatory Network

The Circular RNA Interactome (CircInteractome) (https://circinteractome.nia.nih.gov/) and Cancer-Specific CircRNA (CSCD) (http://gb.whu.edu.cn/CSCD/) were used to predict miRNA binding sites (MREs). These miRNAs were considered potential target miRNAs of the DEcircRNAs. DEmiRNA further screened these target miRNAs based on the TCGA.

Interactions between miRNA and mRNA were predicted based on the TargetScan [14], miRTarBase [15], and miRDB [16] databases. Only mRNAs recognized by all three databases were considered candidate mRNAs and intersected with DEmRNAs to screen the DEmRNAs targeted by DEmiRNAs. The circRNA-miRNA-mRNA regulatory network was constructed using a combination of circRNA–miRNA pairs and miRNA–mRNA pairs. Finally, the network was visualized and mapped using Cytoscape v3.7.0 [17].  Figure 1 shows a flow chart for the development of the ceRNA network.

### 2.4. Gene Ontology and Pathway Enrichment Analyses of DEGs in the ceRNA Network

To assess the function of differentially expressed genes (DEGs) in the ceRNA network in tumorigenesis, Gene Ontology (GO) annotation, and Kyoto Encyclopedia of Genes and Genomes (KEGG) pathway analyses were performed using the clusterProfiler package [18] of R software. *P* value < 0.01 was set as the cut-off criterion.

### 2.5. Survival Analysis and Correlation Analysis of DEmiRNAs and DEmRNAs in ceRNA Networks

Each sample in the TCGA was independent of each other and contained all sample information, such as gene expression, prognosis, and survival time. We obtained clinical information from breast cancer patients from the TCGA database and combined the expression data of DEmiRNAs and DEmRNAs with clinical data from patients. A survival package of R was used to perform survival analysis of DEmiRNAs and DE mRNAs in the ceRNA network with *P* < 0.05 used as the threshold. In addition, DEmiRNAs and DEmRNAs with significant overall survival were identified as prognostic biomarkers.

In the TCGA-BRCA dataset, the vast majority of samples were present in both miRNA and mRNA expression profiles, and samples that were only present in one expression profile were deleted. Correlation analysis between the interacting miRNA and mRNA in the ceRNA network was performed using R software, with *r* < −0.3, *P* < 0.001 as the threshold. The miRNA–mRNA pair that satisfied the condition was considered to have a strong negative correlation.

### 2.6. Construction PPI Network and Module Analysis

To assess the interactions between the DEGs in the ceRNA network, we constructed a protein-protein interaction (PPI) network using the Search Tool for the Retrieval of Interacting Genes (STRING, http://string.embl.de/) online tool. We used the MCODE plugin to screen modules of hub genes from the PPI network. The interaction network was visualized using Cytoscape software.

### 2.7. Quantitative Real-Time PCR Validation

Ten pairs of breast cancer tissues and corresponding adjacent nontumor tissues from BRCA patients were obtained from the Department of Breast Disease, The First Affiliated Hospital of Jiaxing University. The study was approved by the ethics committee, and written informed consent was obtained from all patients.

In this ceRNA network, we randomly selected six circRNAs, miRNAs, and mRNAs, respectively, and verified the prediction results' reliability and validity in BRCA patients using qRT-PCR. Total RNA was isolated using TRIzol reagent (Invitrogen, USA) according to the manufacturer's protocol, and RNA purity was detected by NanoDrop 2000 spectrometer (Thermo Fisher Scientific, Waltham, MA, USA). Based on SuperReal PreMix Plus (Invitrogen, USA) in StepOnePlus Real-time PCR Detection System (Applied Biosystems, Foster City, CA, USA), the qRT-PCR reactions were performed. The relative gene expression was calculated by 2^-△△Ct^. The human *β*-actin and human U6 were used as endogenous controls for mRNA and miRNA expressions in analysis, respectively. The human GAPDH was used as endogenous controls for circRNA expression in the analysis.

## 3. Results

### 3.1. Identification of Differentially Expressed RNAs in Breast Cancer

Compared to adjacent tissues, a total of 2762 DEmRNAs (1118 upregulated and 1644 downregulated miRNAs) and 158 DEmiRNAs (71 upregulated and 87 downregulated miRNAs) were identified in BRCA with FDR < 0.01 and ∣log_2_fold change | >1. A total of 72 DEcircRNAs (51 upregulated and 21 downregulated circRNAs) were obtained in BRCA compared to adjacent tissues with *P* value < 0.01, ∣log_2_fold change | >1. The RNA hierarchical clustering analyses are presented in Figure 2. It was demonstrated that the expression levels of these three types of RNAs were significantly differentiated compared with the normal tissues. Finally, volcano plots were generated, and differences between the normal and tumor groups were identified (Figure 2). Supplementary table 1, 2, and 3 show the top 10 up- and downregulation of DEmRNAs, DEmiRNAs, and DEcircRNAs in BRCA, respectively.

### 3.2. Construction of ceRNA Regulatory Network in BRCA

To elucidate the regulatory mechanism of BRCA, a circRNA-miRNA-mRNA-related ceRNA network of BRCA was developed according to the above results. First, we searched for the target miRNAs of the 72 DEcircRNAs in the CircIteractome and CSCD databases and found 295 interactive circRNA–miRNA pairs after intersecting with the DEmiRNAs. The circRNA–miRNA relationship pairs were screened according to a negative regulatory pattern and positively coexpressed circRNA–miRNA pairs were discarded. The results showed that 162 interactive circRNA–miRNA pairs were screened, of which 72 DEmiRNAs were confirmed to interact with 59 DEcircRNAs. Following this, we predicted that 1626 mRNAs were targeted by these 72 DEmiRNAs in all three target predicting databases (TargetScan, miRTarBase, and miRDB). These 1626 target mRNAs intersected with the 2762 DEmRNAs, and target mRNAs not contained in DEmRNAs were excluded, resulting in 327 interactive miRNA–mRNA pairs. At the same time, we also screened miRNA–mRNA pairs based on negative regulatory patterns and discarded positively coexpressing pairs. The results showed that eventually, 30 DEmiRNAs and 100 DEmRNAs formed 140 interactive miRNA–mRNA pairs. The circRNA–miRNA and miRNA–mRNA relationship pairs (Supplementary tables 4 and 5) were combined into the ceRNA network following the pattern of negative regulation. Finally, we constructed the ceRNA regulatory network of BRCA comprised of 200 edges among 40 DEcircRNAs, 30 DEmiRNAs, and 100 DEmRNAs. The ceRNA network in BRCA was visualized using Cytoscape software (Figure 3).

### 3.3. Functional Annotation of the DEGs in the ceRNA Network

In order to better understand the potential functional significance of differentially expressed genes in the ceRNA network, GO and KEGG functional enrichment analyses were performed. In the GO analysis, we identified 162 enriched GO terms (FDR < 0.01). The top 8 significantly enriched GO terms in the biological process (BP), cellular components (CC), and molecular function (MF) are shown in Figure 4. The biological processes of these differentially expressed genes were primarily involved in protein kinase B signaling, phosphatidylinositol phosphorylation, protein kinase B signaling, and lipid phosphorylation. Meanwhile, the genes related to cellular components were mostly involved in nuclear transcription factor complex, focal adhesion, cell-substrate adherens junction, and cell-substrate junction. In terms of molecular function, these differential genes were mostly enriched in phosphatidylinositol-4,5-bisphosphate 3-kinase activity, phosphatidylinositol bisphosphate kinase activity, phosphatidylinositol 3-kinase activity, and 1-phosphatidylinositol-3-kinase activity.

Additionally, KEGG signal pathway analysis showed that 24 signal pathways were significantly enriched (FDR < 0.01). The top 15 significantly enriched pathways are shown in Figure 5. Among these pathways, the ‘PI3K-Akt signaling pathway,' ‘MicroRNAs in cancer,' ‘Proteoglycans in cancer,' ‘Cellular senescence,' ‘FoxO signaling pathway,' ‘Central carbon metabolism in cancer,' and ‘Cell cycle' are closely correlated with the carcinogenesis and development of BRCA.

### 3.4. Prognostic Characteristics of RNAs in the ceRNA Regulatory Network

Survival analysis based on the Survival package of R found that 13 mRNAs (CCNE1, TPD52, SDC1, ANLN, ZNF367, SOX11, IRS2, EZR, DSC3, CCND2, KPNA2, CBX2, and CEP55) among the 100 DEmRNAs in the ceRNA network were closely associated with the overall survival of breast cancer patients. The low expression of CCNE1, TPD52, SDC1, ANLN, ZNF367, SOX11, EZR, KPNA2, CBX2, and CEP55 was associated with high survival, whereas for IRS2, DSC3, and CCND2, high expression was associated with high survival. Six miRNAs (hsa-miR-204-5p, hsa-miR-335-5p, hsa-miR-100-5p, hsa-miR-195-5p, hsa-miR-328-3p, and hsa-miR-342-3p) of 30 DEmiRNAs were associated with prognosis. High expression of hsa-miR-204-5p, hsa-miR-335-5p, hsa-miR-100-5p, hsa-miR-195-5p, and hsa-miR-342-3p indicated long survival time, while high expression of hsa-miR-328-3p indicated a relatively short survival time. Survival analysis results are shown in Table 1 and Figure 6. Notably, based on the ceRNA network, we found that the hsa_circ_0004315-hsa-miR195-5p axis was associated with four mRNAs associated with breast cancer prognosis.

### 3.5. Interaction between miRNA and mRNA from the ceRNA Network

According to the ceRNA theory, circRNA could indirectly affect mRNA through miRNA. At the expression level, miRNA was negatively correlated with circRNA and mRNA. To verify that the network we built was consistent with ceRNA theory, we performed the correlation analysis on different kinds of RNA. The expression information of circRNA in this study was from the GSE101123 dataset, while the expression information of miRNA and mRNA were from the TCGA dataset. Since RNAs' expression information in the correlation analysis must be from the same sample, this study could only analyze the correlation between miRNA and mRNA expression levels. We performed a correlation analysis of miRNA–mRNA pairs in the ceRNA network based on R software, and the results showed that there were 48 miRNA-mRNA pairs with a strong negative correlation (*r* < −0.3, *P* < 0.001) (Table 2). For instance, hsa-miR-141-3p negatively correlated with ZEB2 (*r* = −0.599, *P* < 0.001) and QKI (*r* = −0.535, *P* < 0.001), hsa-miR-195-5p negatively correlated with CEP55 (*r* = −0.547, *P* < 0.001) and CLSPN (*r* = −0.525, *P* < 0.001), and hsa-miR-200a-3p negatively correlated with ZEB2 (*r* = −0.520, *P* < 0.001) as well as QKI (*r* = −0.513, *P* = 0.001) (Figure 7).

### 3.6. Construction of PPI Network and Module Analysis

The STRING database was used to unveil the interrelationships between the DEmRNAs in the ceRNA network by constructing a PPI network. This PPI network involves 75 nodes and 283 edges. Visualization was performed with Cytoscape (Figure 8(a)). In order to identify hub genes in the process of BRCA carcinogenesis, the MCODE plugin in Cytoscape was used to identify the core subnetwork in the PPI network. Two core subnetworks were obtained, including 21 genes and 49 edges (Figure 8(b)). We used these 21 genes as potential hub genes.

### 3.7. Quantitative Real-Time PCR Validation

Finally, we randomly selected four DEcircRNAs, DEmiRNAs, and DEmRNAs, respectively, in the ceRNA network to verify the above analysis results' reliability and validity. These results showed that CCNE1, CEP55, ANLN, hsa-miR-592, hsa-miR-141-3p, hsa_circ_0000069, hsa_circ_0000518, and has_circ_0000520 were upregulated in BRCA tumor tissues compared to adjacent nontumor tissues, while ADIPOQ, hsa-miR-195-5p, hsa-miR-204-5p, and has_circ_0000977 were downregulated in BRCA tumor tissues (Figure 9). The results of qRT-PCR validation from new breast cancer patients were consistent with the above bioinformatics results, indicating that our bioinformatics analysis was credible.

## 4. Discussion

Abnormal expression of circRNA has been widely observed in various diseases. Studies have shown that dysregulated circRNA has a key role in cancer [19]. However, only a few studies have described the profile of circRNA in BRCA by microarray analysis. The constructed BRCA-related circRNA-associated ceRNA network provides important hints for detecting the key RNAs of the ceRNA-mediated gene regulatory network in the initiation and development of BRCA.

We obtained BRCA mRNA, miRNA expression profile, and circRNA expression profile from the TCGA and GEO databases. After statistical analysis, 2762 DEmRNAs, 158 DEmiRNAs, and 72 DEcircRNAs were identified. Next, we screened the circRNA–miRNA interaction pairs through CircIteractome and CSCD databases, screened the miRNA–mRNA interaction pairs by TargetScan, miRTarBase, and miRDB databases and then took the intersection and finally constructed a specific circRNA-miRNA-mRNA ceRNA regulatory network. We have found that specific circRNAs in this ceRNA network, such as hsa_circ_0000376, hsa_circ_0000069, hsa_circ_0000520, hsa_circ_0008365, and hsa_circ_0000511 have also been reported as potential diagnostic markers in certain cancers. hsa_circ_0000376 is highly expressed in gastric cancer tissues [20], and there are reports that it is involved in the occurrence of breast cancer [21]. hsa_circ_0000069 is upregulated in colorectal cancer tissues, which can promote the proliferation, migration, and invasion of tumor cells [22]. hsa_circ_0000520 was upregulated in breast cancer and cell lines (T47D, MCF-7, MDA-MB-231, BT549, and SKBR3), and hsa_circ_0000520 high expression was associated with poor overall survival [23]. hsa_circ_0008365 (circ-SERPINE2) is a novel proliferative promoter that can regulate YWHAZ through sponge miR-375 to promote the development of gastric cancer [24]. The knockdown of has_circ_0000069 can inhibit the occurrence of pancreatic cancer and may be a potential target for the treatment of pancreatic cancer [25] hsa_circ_0000511 improves epithelial mesenchymal transition in cervical cancer by targeting hsa-miR-296-5p/HMGA1 axis, which is consistent with the ceRNA axis found in this study [26].

We performed GO analysis and KEGG analysis to understand the potential functional significance of differentially expressed mRNA in ceRNA networks. KEGG analysis found that some enriched signaling pathways were closely related to the development of cancer, such as ‘PI3K-Akt signaling pathway' [27], ‘MicroRNAs in cancer,', ‘Proteoglycans in cancer,' ‘Cellular senescence,' ‘FoxO signaling pathway' [28], ‘Central carbon metabolism in cancer,' and ‘Cell cycle' [29]. Functionally annotated results also indicate that circRNAs, which regulate these key mRNAs, may have an important role in initiating and developing BRCA and pathways associated with cancer genes.

To further identify the key genes involved in the regulatory network, we established a PPI network and screened two core subnetworks through the MCODE plug-in, which contained 21 genes used as potential hub genes. At the same time, we analyzed the relationship between DEmRNAs and DEmiRNAs in ceRNA networks and the overall survival of breast cancer patients. Our results revealed that 13 mRNAs (CCNE1, TPD52, SDC1, ANLN, ZNF367, SOX11, IRS2, EZR, DSC3, CCND2, KPNA2, CBX2, and CEP55) and 6 miRNAs (hsa-miR-204-5p, hsa-miR-335-5p, hsa-miR-100-5p, hsa-miR-195-5p, hsa-miR-328-3p, and hsa-miR-342-3p) were significantly associated with the prognosis of breast cancer patients. Most of these molecules related to patient survival are thought to be related to the molecular pathogenesis of various tumors and were closely related to the occurrence, development, proliferation, metastasis, and prognosis of cancer [30–34]. For example, the DNA copy number of TPD52 is amplified in prostate cancer cells, and the level of TPD52 protein may be regulated by androgen. Previous studies have shown that genomic amplification and dysregulation of TPD52 caused by androgen induction may have a role in prostate cancer development [31]. Furthermore, Cui et al. found that SDC1 is overexpressed in breast cancer and may be a potential prognostic indicator for breast cancer [32]. Moreover, it has been reported that the upregulation of ANLN is a common feature in the carcinogenesis of lung tissue. ANLN can have a key role in developing human lung cancer by activating RHOA and participating in the phosphoinositide 3-kinase/AKT pathway. Also, the expression of ANLN is associated with low survival in patients with NSCLC [33]. CEP55 is a determinant of mitosis in breast cancer cells [34]. Additionally, it was found that EZR is upregulated in breast cancer and can be used as a potential marker for breast cancer's overall survival [35]. Li et al. found that hsa-miR-195-5p can be used as a biomarker for the diagnosis of lung cancer [36]. hsa-miR-204-5p can be used as a potential prognostic marker and therapeutic target in thyroid cancer [37].

It is well known that miRNAs regulate about 60% of human genes and mediate various biological pathways, including pathways critical for tumorigenesis. Herein, we found that microRNAs associated with BRCA overall survival in ceRNA networks had an important role in tumorigenesis, development, prognosis, and drug resistance. Extracellular vesicles containing miR-335-5p can reduce the growth and invasion of liver cancer *in vitro* and *in viv*o, suggesting that exosome miR-335-5p can be used as a novel therapeutic strategy for hepatocellular carcinoma [38]. Nabavi et al. identified miR-100-5p as one of the key molecular components in the initiation and evolution of androgen ablation therapy resistance in prostate cancer [39]. Moreover, a research team reported that miR-328-3p is upregulated in ovarian cancer stem cells (CSC). A high expression of miR-328-3p can directly target DNA damage-binding protein 2 to maintain CSC properties. The inhibition of miR-328-3p is a new strategy that can effectively eliminate CSC [35]. Enhanced expression of miR-342-3p synergizes with miR-205-5p to inhibit E2F1, thereby reducing tumor chemoresistance [40]. In addition, studies have shown that hsa-miR-204-5p can be used to predict the prognosis of patients with clear renal cell carcinoma, lung adenocarcinoma, and other cancers [41, 42]. hsa-miR-204-5p directly targets FOXA1 to regulate tumor cell infiltration and metastasis [43] and can affect tumor angiogenesis by interfering with the expression of ANGPT1/TGFBR2 [44]. hsa-miR-195-5p can affect colorectal cancer development by inhibiting the Hippo-YAP pathway [45]; meanwhile, hsa-miR-195-5p can be used as a potential diagnostic and prognostic target in breast cancer [46].

We performed a correlation analysis between the expression levels of miRNAs and mRNAs from the same sample in the TCGA database. The results revealed 43 pairs of interconnected miRNAs and mRNAs with a significant negative correlation in the constructed miRNA–mRNA interaction pairs. These links have also been found in some reports. For example, Luo et al. found that overexpression of hsa-miR-195-5p can reduce the expression level of CCNE1. Targeting this miRNA may be used as a new strategy for diagnosing and treating breast cancer [46]. In addition, reports on circRNA found that circAGFG1 can act as a sponge of hsa-miR-195-5p, which promotes triple-negative breast cancer by regulating the expression of CCNE1 [47]. These results also indirectly reflect the feasibility of using bioinformatics to construct regulatory networks. At the same time, we collected clinical breast cancer samples and verified by fluorescence quantitative PCR for some differentially expressed molecules, which is consistent with the results of our analysis. This also shows the credibility of our results.

This study is aimed at exploring new therapeutic targets and biomarkers for breast cancer by constructing circRNA-related ceRNA networks. However, most of the results of this study are derived from bioinformatics analysis. The physiological mechanism of the selected differential molecules and their potential as breast cancer biomarkers need to be further studied. There are some shortcomings here. First of all, there are too few samples included in this study to draw clear conclusions. Secondly, the role of these randomly verified differential molecules in breast cancer is still not very clear, and further functional exploration is needed. Finally, this study only verified a small number of differential molecules. If all differential molecules can be verified, it is possible to obtain a more accurate and reliable ceRNA network. In the future, more samples and more studies are needed to verify these conclusions.

## 5. Conclusion

This study identified unusually expressed key RNAs by analyzing the RNA expression profiles of BRCA in public databases. This specific circRNA, miRNA, and mRNA molecules may help discover sensitive biomarkers in BRCA. More importantly, we have constructed a circRNA-miRNA-mRNA ceRNA network that will be used to elucidate the unknown ceRNA regulatory axes in BRCA. Our findings provide novel insights into an in-depth understanding of circRNA-related ceRNA networks in breast cancer as well as potential diagnostic and prognostic biomarkers.

## Figures and Tables

**Figure 1:** Flow chart of comprehensive bioinformatics analysis in constructing competing endogenous RNA (ceRNA) regulatory network.

**Figure 2:** Heatmap and volcano diagrams of breast cancer-related differentially expressed mRNAs, miRNAs, and circRNAs. (a) mRNA. (b) miRNA. (c) circRNA. The color from blue to red shows a trend from low expression to high expression. The red dot represents upregulated mRNA, miRNA, and circRNA; the green dot represents downregulated mRNA, miRNA, and circRNA.

**Figure 3:** Competing endogenous RNA (ceRNA) (DEcircRNA-DEmiRNA-DEmRNA) regulatory network. The v nodes, round rectangle nodes, and elliptical nodes indicate DEcircRNAs, DEmiRNAs, and DEmRNAs, respectively. Red and blue represent upregulation and downregulation, respectively. Green borders surrounding the nodes indicate prognostic significance. Purple edges indicate a good negative correlation between RNAs.

**Figure 4:** Significantly enriched Gene Ontology (GO) terms of differentially expressed mRNAs in the ceRNA regulatory network. BP: biological process; CC: cellular component; MF: molecular function. The *x*-axis shows counts of host genes enrich in GO terms, and the *y*-axis shows GO terms. The color scale represented *P*.adjust.

**Figure 5:** Significantly enriched the Kyoto Encyclopedia of Genes and Genomes (KEGG) pathways of differentially expressed mRNAs in the ceRNA regulatory network. The *x*-axis shows counts of host genes enrich in KEGG pathways, and the *y*-axis shows KEGG pathways. The color scale represented *P*.adjust.

**Figure 6:** Kaplan-Meier survival curves of differentially expressed miRNAs (DEmiRNAs) and differentially expressed mRNAs (DEmRNAs) in the competing endogenous RNA (ceRNA) network that is significantly associated with overall survival in breast cancer.

**Figure 7:** Pearson's correlation analysis between the interacting miRNA and mRNA expression in the ceRNA network.

**Figure 8:** Identification of hub genes from the PPI network with the MCODE algorithm. (a) PPI network construction. (b) Two core subnets with 21 hub genes. Red nodes represent the upregulated genes; blue nodes represent downregulated genes. PPI: protein-protein interaction.

**Figure 9:** qRT-PCR validation of the DEmRNAs, DEmiRNAs, and DEcircRNAs in breast cancer. The *x*-axis represents the DEmRNAs/DEmiRNAs/DEcircRNAs, and the *y*-axis represents log_2_(fold change).

**Table 1:** Prognostic value of the differentially expressed mRNAs and miRNAs.

Name	HR (95% CI)	*P* value
CCNE1	1.606 (1.169-2.208)	0.0038
TPD52	1.578 (1.148-2.169)	0.0053
SDC1	1.516 (1.102-2.086)	0.0102
ANLN	1.489 (1.083-2.046)	0.0154
ZNF367	1.475 (1.073-2.025)	0.0176
SOX11	1.443 (1.050-1.983)	0.0244
IRS2	0.705 (0.512-0.971)	0.0299
EZR	1.418 (1.030-1.950)	0.0311
DSC3	0.718 (0.521-0.988)	0.0398
CCND2	0.718 (0.522-0.987)	0.0400
KPNA2	1.395 (1.015-1.917)	0.0410
CBX2	1.391 (1.012-1.912)	0.0433
CEP55	1.384 (1.007-1.902)	0.0474
hsa-miR-195-5p	0.629 (0.455-0.870)	0.0046
hsa-miR-204-5p	0.648 (0.469-0.894)	0.0086
hsa-miR-335-5p	0.664 (0.481-0.916)	0.0134
hsa-miR-342-3p	0.696 (0.504-0.961)	0.0280
hsa-miR-100-5p	0.704 (0.509-0.972)	0.0323
hsa-miR-328-3p	1.410 (1.021-1.947)	0.0356

**Table 2:** Correlation analysis of the relationship between miRNA and mRNA.

miRNA	mRNA	*R*	*P* value
hsa-miR-141-3p	ZEB2	-0.59875	0
hsa-miR-195-5p	CEP55	-0.54744	0
hsa-miR-141-3p	QKI	-0.53509	0
hsa-miR-195-5p	CLSPN	-0.52524	0
hsa-miR-200a-3p	ZEB2	-0.52049	0
hsa-miR-200a-3p	QKI	-0.51254	0
hsa-miR-195-5p	HMGA1	-0.49915	0
hsa-miR-497-5p	CEP55	-0.49525	0
hsa-miR-195-5p	CHEK1	-0.49341	0
hsa-miR-195-5p	CDC25A	-0.49147	0
hsa-miR-195-5p	CCNE1	-0.48761	0
hsa-miR-497-5p	ANLN	-0.45814	0
hsa-miR-139-5p	TPD52	-0.44566	0
hsa-miR-195-5p	E2F7	-0.44235	0
hsa-miR-139-5p	ZNF367	-0.43672	0
hsa-miR-497-5p	CLSPN	-0.43102	0
hsa-miR-145-5p	TPM3	-0.42875	0
hsa-miR-195-5p	CBX2	-0.42701	0
hsa-miR-145-5p	RTKN	-0.42632	0
hsa-miR-195-5p	ZNF367	-0.42269	0
hsa-miR-200a-3p	DLC1	-0.4224	0
hsa-miR-497-5p	CCNE1	-0.42016	0
hsa-miR-7-5p	RBMS3	-0.41862	0
hsa-miR-497-5p	CDC25A	-0.4139	0
hsa-miR-342-3p	ID4	-0.4063	0
hsa-miR-497-5p	CHEK1	-0.40444	0
hsa-miR-141-3p	STAT5A	-0.39451	0
hsa-miR-218-5p	LMNB1	-0.3945	0
hsa-miR-141-3p	YAP1	-0.3803	0
hsa-miR-497-5p	CBX2	-0.37969	0
hsa-miR-200a-3p	HGF	-0.37823	0
hsa-miR-497-5p	E2F7	-0.3743	0
hsa-miR-218-5p	TPD52	-0.37324	0
hsa-miR-195-5p	CDCA4	-0.3683	0
hsa-miR-204-5p	AP1S1	-0.36607	0
hsa-miR-497-5p	CDCA4	-0.36528	0
hsa-miR-204-5p	EZR	-0.35209	0
hsa-miR-497-5p	ZNF367	-0.34916	0
hsa-miR-7-5p	SNCA	-0.33958	0
hsa-miR-145-5p	ABRACL	-0.33926	0
hsa-miR-365b-3p	MCOLN2	-0.33306	0
hsa-miR-365a-3p	MCOLN2	-0.33285	0
hsa-miR-141-3p	USP53	-0.31765	0
hsa-miR-200a-3p	YAP1	-0.3142	0
hsa-miR-145-5p	ABHD17C	-0.3107	0
hsa-miR-33b-5p	GAS1	-0.3097	0
hsa-miR-195-5p	ENTPD7	-0.30541	0
hsa-miR-33b-5p	ARID5B	-0.3005	0

## Data Availability

The data used to support the findings of this study are available from the corresponding author upon request.

## Supplementary Materials

Supplementary Materials Supplementary Table 1: top 10 upregulation and downregulation DEmRNAs in BRCA. Supplementary Table 2: top 10 upregulation and downregulation DEmiRNAs in BRCA. Supplementary Table 3: top 10 upregulation and downregulation DEcircRNAs in BRCA. Supplementary Table 4: interaction between circRNA and miRNA in the ceRNA network. Supplementary Table 5: interaction between miRNA and mRNA in the ceRNA network.
